# Prevalence of Urinary Tract Infection and Its Associated Factors among Pregnant Women in Ethiopia: A Systematic Review and Meta-Analysis

**DOI:** 10.1155/2021/6551526

**Published:** 2021-12-01

**Authors:** Temesgen Getaneh, Ayenew Negesse, Getenet Dessie, Melaku Desta, Agimasie Tigabu

**Affiliations:** ^1^Department of Midwifery, College of Health Science, Debre Markos University, Debre Markos, Ethiopia; ^2^Department of Human Nutrition and Food Science, College of Health Science, Debre Markos University, Debre Markos, Ethiopia; ^3^Center of Excellence in Human Nutrition, School of Human Nutrition, Food Science and Technology, Hawassa University, Ethiopia; ^4^Department of Nursing, College of Medicine and Health Science, Bahir Dar University, Bahir Dar, Ethiopia; ^5^Department of Nursing, College of Health Science, Debre Tabor University, Debre Tabor, Ethiopia

## Abstract

**Objective:**

Urinary tract infection (UTI) is the most common bacterial infections during pregnancy. It is associated with different maternal and neonatal adverse outcomes such as low birth weight, preterm birth, still birth, preeclampsia, maternal anemia, sepsis, and amnionitis, even when the infection is asymptomatic. However, in Ethiopia, it is represented with fragmented and inconclusive pocket studies. Therefore, this systematic review and meta-analysis is aimed at estimating the pooled prevalence of UTI and its associated factors among pregnant women in Ethiopia.

**Methods:**

PubMed/Medline, Embase, Cochrane Library, Google Scholar, and local sources were used to access eligible studies. Joanna Briggs Institute Meta-Analysis of Statistics Assessment and Review Instrument was applied for critical appraisal. Heterogeneity and publication bias were evaluated using *I*^2^ statistic, funnel plot asymmetry, and Egger's tests. Random effect model was employed to estimate the pooled burden of UTI and its associated factors among pregnant women with its corresponding odds ratio (OR) and 95% confidence interval (CI).

**Result:**

From all systematically searched articles, 14 studies were eligible for this analysis. The overall pooled prevalence of UTI among pregnant women in Ethiopia was 15.37% (95% CI: 12.54, 18.19). Family monthly income (OR = 3.8 and 95% CI: 1.29, 11.23), parity (OR = 1.59 and 95% CI: 1.01, 2.50), history of catheterization (OR = 2.76 and 95% CI: 1.31, 5.84), and history of UTI (OR = 3.12 and 95% CI: 1.74, 5.60) were factors significantly associated with UTI among pregnant women in Ethiopia.

**Conclusion:**

The overall pooled estimate of UTI among pregnant women in Ethiopia was higher compared with CDC estimation which was 8%. Family monthly income < 1000ETB, multipara, previous history of catheterization, and history of UTI were factors increased burden of UTI during pregnancy. So, strategies targeting in economic reforms, universal access of family planning, and standardized prenatal care service should be addressed to alleviate this high prevalence of UTI during pregnancy.

## 1. Introduction

The likelihood of urinary tract infections (UTIs) is increased during pregnancy due to numerous women's physiological changes [1]. The main reason is due to urinary stasis and vesicoureteral reflux caused by hormonal and mechanical changes [2]. In addition, short urethra and difficulty with hygiene due to a distended pregnant belly make UTI the commonest bacterial infectious during pregnancy which occurs in about 8% of pregnant women [3]. Furthermore, pregnant patients are considered immunocompromised UTI hosts because of the physiologic changes associated with pregnancy [4]. These changes increase the risk of serious infectious complications from symptomatic and asymptomatic urinary infections even in healthy pregnant women [5].

It is associated with increased risks of maternal and neonatal morbidity and mortality, even when the infection is asymptomatic [6]. If asymptomatic bacteriuria is untreated in pregnancy, the rate of subsequent UTI is approximately 25% [6]. Even though maternal UTI has few direct fetal sequelae because fetal bloodstream infection is rare, uterine hypoperfusion due to maternal dehydration, maternal anemia, and direct bacterial endotoxin damage to the placental vasculature may cause fetal cerebral hypoperfusion [7].

It may also pose a serious health risk to a pregnant woman and developing fetus and cause of antepartum intensive care unit admission [8]. It is associated with different maternal and neonatal adverse outcomes such as low birth weight, premature labor and prematurity, still birth, preeclampsia, maternal anemia and sepsis, and amnionitis [9, 10]. In addition, it is also associated with premature rapture of membrane and low Apgar score. This may lead to increased maternal and perinatal morbidity and mortality [11, 12]. Furthermore, UTI during pregnancy is independently associated with intrauterine growth restriction, preeclampsia, preterm delivery, and cesarean delivery [13, 14]. In addition to those adverse risks, it also had financial threats in which the annual health costs for UTI exceed two billion$. Screening for these conditions in pregnant women is cost-effective, compared with treating UTI and its complication [15].

Evidences showed that pregnant women in developing countries have higher rates of UTI and its burden than developed nations [5, 16]. Previous history of UTI, preexisting diabetes, increased parity, low socioeconomic status, immunosuppression, tobacco use, extreme maternal age, and late presentation for prenatal care are some of the risk factors [17, 18]. Among the common cause of UTI during pregnancy, Escherichia coli shared the highest while the rest was caused by different pathogens like Klebsiella pneumoniae, Proteus mirabilis, Enterobacter species, Staphylococcus saprophytic, and group B beta hemolytic streptococcus [7].

In Ethiopia, the burden of UTI among pregnant women widely varies. It ranges from 9.8% [19] to 26.6% [20]. Several fragmented individual studies were done in Ethiopia to estimate the show of the burden of UTI and its associated factors among pregnant women [19–33]. Among these studies, the lowest burden of UTI was reported in Amhara region [19] while the highest burden was occurred in Oromo regional state of Ethiopia [20]. Furthermore, sociodemographic factors like maternal age, residence, marital status, maternal educational status, monthly family income, and maternal occupation and medical and obstetric related factors like anemia, HIV status, history of UTI, history of catheterization, parity, and gestational age were some of modifiable and nonmodifiable factors stated in each fragmented studies as a potential-associated factors for UTI among pregnant women in Ethiopia [19, 21, 22, 25–27, 31, 32]. However, all of these studies were inconclusive. Currently in Ethiopia, there is no concrete evidence reporting the overall pooled prevalence of UTI and its associated factors among pregnant women. Therefore, this systematic review and meta-analysis was aimed at estimating the pooled prevalence of UTI and its associated factors among pregnant women in Ethiopia.

## 2. Methods

### 2.1. Searching Strategies

From Prospero, burden of UTI and its associated factors among pregnant women in Ethiopia: systematic review and meta-analysis was searched to avoid duplication. To the best of our knowledge, this is the first systematic review meta-analysis done in Ethiopia in this title. PubMed, Medline, Embase, Cochrane Library, Google Scholar, and local sources including academic and governmental institution online library were used to access included articles. In addition, the cross-references (lists of already identified articles references) were applied to retrieve studies. The key terms used for systematically searching relevant literatures were UTI, asymptomatic or symptomatic, bacteriuria, bacteria profile, prenatal, pregnancy, antenatal, associated factors, determinants, predictors, risk factors, causes, and Ethiopia. All studies on electronic databases and local sources were searched till March/2021. Then, identified articles were exported into endnote citation manager software version X7 for Windows to exclude duplicate records. The Preferred Reporting Items for Systematic Reviews and Meta-Analyses Protocols (PRISMA) checklist guidelines [34] were used to develop this systematic review and meta-analysis.

### 2.2. Eligibility Criteria

*Study scope*: all studies conducted in all regional states and administrative cities of Ethiopia on burden of UTI and its associated factors during pregnancy were included under this systematic review and meta-analysis. No restriction was applied to language, study design, study setting, and publication.

*Population*: all reproductive aged women (15-49 years) who were pregnant at least once were considered for this review.

*Exposure*: all studies explored burden of UTI and its associated factors among pregnant women in Ethiopia were included.

*Outcome variable*: studies which diagnosed UTI during pregnancy when their urine yielding positive cultures (≥10^5^ CFU/ml) were included for this review.

After all identified studies title and abstract screened for eligibility, studies unrelated to our review title were excluded. Then, full texts of those articles related to our title and eligible were critically examined. However, those papers which did not fully access at the time of our search process were excluded after contact was attempted with the principal investigator through email at least two times. Furthermore, after reviewing full texts of all eligible studies, studies which did not report our outcome of interest and studies with poor quality as per settled criteria of reviewing the articles were excluded from the final analysis.

### 2.3. Data Extraction

Data extraction was undertaken using standardized data extraction Excel spreadsheet format prepared according to 2014 Joanna Briggs Institute Reviewers' Manual [35]. This standardized data extraction format includes the following: author name, study of region, publication year, study design, sampling technique, study setting, sample size, mean age of respondent, standard used to diagnosed UTI, response rate, and prevalence of UTI among pregnant women. Factors associated with UTI during pregnancy were also systematically extracted using cross tabulation between UTI and those potential-associated factors (including sociodemographic factors like maternal age (≥25 yrs vs. <25 yrs), residence (rural vs. urban), marital status (married vs. single), maternal educational status (illiterate vs. formal education), monthly family income (<1000ETB vs. ≥1000ETB in which 1000ETB is equivalent with 23.8$ and we have used the cut point 1000ETB because the exist data were not classified based similarly and not based on national income level classification), and maternal occupation (housewife vs. employed)) and medical and obstetric related factors like anemia (yes vs. no), HIV status (positive vs. negative), history of UTI (yes vs. no), history of catheterization (yes vs. no), parity (multipara vs. primipara and nulliparous), and gestational age (second and third trimester vs. first trimester). Disagreements between the authors were resolved by face to face discussion and consensus.

### 2.4. Quality Assessment

Before data extraction was handled, critical appraisal of included and eligible studies was employed using Joanna Briggs Institute Meta-Analysis of Statistics Assessment and Review Instrument (JBI-MAStARI) [35]. In the appraisal tool, randomness of subject selection, clear definition of inclusion criteria, identification and addressing for confounding factors, clear objective, and reliable measurement of outcome variable and use of appropriate statistical analysis method were included. Two independent reviewers evaluated each included individual studies critically. Disagreements between the reviewers were resolved via discussion and consensus. If not, the third reviewer was involved. Finally, those articles scored five and above were considered in this review.

We assessed and evaluated the methodological quality and risk of bias in the studies that were selected using the 10-item rating scale developed by Hoy et al. for prevalence studies [36]. Sampling, data collection, reliability and validity of study tools, case definition, and prevalence periods were included in the tool. The rating scale was categorized as having low risk of bias (“yes” answers to domain questions) or high risk of bias (“no” answers to domain questions) for each articles. Each study was assigned a score of 1 (yes) or 0 (no) for each domain, and these scores were summed to provide an overall study quality score. Scores of 8-10 were considered as having a “low risk of bias,” 6–7 a “moderate risk,” and 0–5 a “high risk.” For the final risk of bias classification, disagreements between the reviewers were resolved via consensus.

### 2.5. Outcome Measurement

The primary outcome of this systematic review and meta-analysis was estimating the pooled burden of UTI among pregnant women in Ethiopia. UTI during pregnancy was diagnosed when their midstream urine sample yields positive cultures (≥10^5^ CFU/ml) in either symptomatic or asymptomatic pregnant women. In addition, this review is also aimed at identifying factors associated with the pooled burden of UTI during pregnancy. Generally, sociodemographic factors like maternal age, residence, marital status, maternal educational status, monthly family income, and maternal occupation and medical and obstetric related factors like anemia, HIV status, history of UTI, history of catheterization, parity, and gestational age were identified factors to be associated with burden of UTI.

### 2.6. Statistical Analysis

Those data extracted using the prepared Excel spreadsheet format were imported to Stata version 14 for further analysis. The existence of heterogeneity was assessed using the Cochran's *Q* statistic while the inverse variance (*I*^2^) was used to quantify it. A value at 25%, 50%, and 75% was considered as low, moderate, and high heterogeneity across studies, respectively [37]. In addition, Egger's regression test and asymmetry funnel plot were applied to assess publication bias [38]. Furthermore, *p* value less than 0.05 was used to declare the presence of heterogeneity across studies and publication bias. Random effect model was computed to estimate the pooled burden of UTI and its associated factors during pregnancy using forest plot diagram with their corresponding 95% CI and OR. Moreover, subgroup analysis and metaregression were conducted to explore potential sources of heterogeneity across studies using different characteristics of the studies. Generally, the methodology part of our research may be overlapped with our previous work which was unpublished (leave for further updating and overall changing) [39].

## 3. Results

### 3.1. Explanation for Original Studies

From medical-related electronic databases and local sources, a total of 245 articles were accessed. 75 articles were excluded because of duplication, and 124 were removed as reason of inconsistent with our review. Then, the remaining 46 studies were assessed and screened based on eligibility criteria. After screening, 31 articles were removed because of irrelevancy. Using JBI-MAStARI, 15 full articles were critical appraised. After critical appraisal, one articles [40] was excluded because of low quality scored. Finally, 14 studies were included for estimating the pooled prevalence of UTI and its associated factors during pregnancy in Ethiopia (Figure 1).

Among 14 eligible and included articles, 12 of them were published studies from 2007 to 2018 whereas the remaining two studies were unpublished. All included articles were conducted using institutional based cross sectional study design. Around 86% of the included studies (12 studies) used consecutive sampling technique while 14% of them (two studies) used systematic random sampling technique. All studies considered UTI among pregnant women when their urine sample yielding positive cultures (≥10^5^CFU/ml) and had 95% and above of response rate. A total of 3,948 reproductive age (15-49) women who have at least one pregnancy were included to estimate the pooled prevalence of UTI and its associated factors during pregnancy in Ethiopia.

From the included studies, six articles were in Amhara regional state [19, 21, 22, 26, 28, 29] whereas Tigray, SNNP and AA shared two articles for each [23, 27, 30–33] while Oromo [20] and Dire Dawa [25] contribute only a single study for each. According to JBI-MAStARI critical appraisal, each included individual articles scored a minimum of five to maximum of 8 out of 9. In addition, nearly 55% of UTI during pregnancy was caused by Gram-negative bacteria (GNB) while the remaining 45% of UTI was caused by Gram-positive bacteria. Furthermore, Escherichia coli is responsible for the cause of around 35% of UTI during pregnancy (Table 1).

In regarding risk bias assessment, 10 (71.5%) studies had high quality scores and 4 (28.5%) had low quality scores (Table 2). Representation and case-definition biases were the most commonly noted. To determine the influence of low methodological quality/high risk of bias on our estimates of pooled prevalence, we estimated pooled prevalence without the low-quality studies. The confidence intervals of our estimates of pooled prevalence with and without these studies overlapped, indicating no significant difference between them. These results suggest that the majority of the primary study authors have met high-quality standards. This lends credibility to our findings.

### 3.2. Prevalence of UTI among Pregnant Women in Ethiopia

The estimating pooled prevalence of UTI among pregnant women in Ethiopia was 15.37% (95% CI: 12.54, 18.19) (Figure 2). The Cochran's *Q* statistic evidenced the presence of moderate statistically significant level of heterogeneity (*I*^2^ = 73.7%, *p* < 0.001) which indicated that the use of random model effect to estimate the pooled prevalence of UTI and its associated factors among pregnant women was appropriate. Therefore, to identify potential sources of heterogeneity, subgroup analysis and metaregression were undertaken. In addition, publication bias was checked using asymmetric funnel plot and Egger's regression test. Both symmetric funnel plot and Egger's test evidenced, and publication bias was not observed in this review (symmetric funnel plot (Figure 3) and Egger's test *p* value = 0.069 (95% CI: 0.201-1.734)).

### 3.3. Subgroup Analysis

Subgroup analysis was also performed using different study characteristics. In regarding to regional burden, more than one-fifth of pregnant women were diagnosed with UTI in SNNP region with prevalence of 22.2% (95% CI: 15, 29). The lowest overall prevalence of UTI among pregnant women was recorded in Amhara regional state of Ethiopia which was 11.6% (95% CI: 9, 13) while in Tigray 16.3% (95% CI: 7, 25) and in AA 13.09% (95% CI: 9, 16) of pregnant women were diagnosed with UTI.

In addition, studies published before 2015 reported 12.2% (95% CI: 9, 15) of UTI among pregnant women whereas studies published after 2015 and after evidenced that 18.8% (95% CI: 13, 23) of UTI among pregnant women. The pooled prevalence of UTI among studies having less 250 sample size was 14.5% (95% CI: 10, 18) whereas studies with sample size of more than 250 indicated 16.4% (95% CI: 11, 21) of UTI among pregnant women (Table 3).

### 3.4. Metaregression

In order to identify potential source of heterogeneity, metaregression was done in addition to subgroup analysis using both continuous and categorical study characteristics. However, none of these variables were found to be statistically significant (Table 4).

### 3.5. Factors Associated with UTI among Pregnant Women in Ethiopia

In addition to estimating the pooled prevalence of UTI among pregnant women in Ethiopia, this review also examined the association of different sociodemographic and medical and obstetric related factors with UTI during pregnancy. Maternal age, residence, marital status, maternal educational status, monthly family income, maternal occupation, anemia, HIV status, history of UTI, history of catheterization, parity, and gestational age were among the factors evaluated. But only monthly family income, history of UTI and catheterization, and parity were significantly associated with the pooled prevalence of UTI among pregnant women (Figures 4–6).

This review showed that monthly family income was significantly associated with UTI among pregnant women in which its association was stated in 6 of the included studies. The odds of UTI among pregnant women with family monthly income less than 1000ETB were 3.8 times higher than their counterparts (OR = 3.8, 95% CI: 1.29, 11.23) (Figure 4).

To evaluate the association between histories of UTI with current UTI among pregnant women, 8 studies were included. The analysis of these studies indicated that the likelihood of UTI among pregnant women who had history of UTI was 3.12 times higher than their counterparts (OR = 3.12, 95% CI: 1.74, 5.60) (Figure 5).

History of catheterization was another significantly associated factor with pooled prevalence of UTI among pregnant women. Its connection with UTI was cited in 7 of included studies. Pregnant women who had history of catheterization were 2.76 times more likely to develop UTI than pregnant women who had no history of catheterization (OR = 2.76, 95% CI: 1.31, 5.84). Once more, parity was also another factor associated with UTI during pregnancy in which its relation was listed in 8 of the original included articles. The odds of UTI among multipara pregnant women were 1.6 times higher than primipara and nulliparous pregnant women (OR = 1.59, 95% CI: 1.01, 2.50) (Figure 6). Maternal age, residence, marital status, maternal educational status, maternal occupation, anemia, HIV status, and gestational age were not associated with pooled burden of UTI among pregnant women in Ethiopia.

## 4. Discussion

This is the first systematic review and meta-analysis done in Ethiopia to estimate the pooled prevalence of UTI and its associated factors among pregnant. According to this review, the overall pooled prevalence of UTI among pregnant women in Ethiopia was 15.37% (95%, CI: 12.54, 18.19). This figure is higher than prevalence of UTI during pregnancy estimated by CDC which was 8%. The possible explanation may be in our country, early initiation of antenatal care service was low. So, there should have early detection and identification of risk factors. In addition, majority of pregnant women will not get health education given for pregnant women for infection prevention due to delay initiation. Furthermore, majority of our population were rural with no formal education which in turn characterize with less level of awareness on infection prevention and health-seeking behavior and lower economic level which will be a significant factor in many aspects.

Therefore, this incompatible and high evidence of the pooled prevalence of UTI during pregnancy in Ethiopia should be taken as a warning and baseline evidence for healthy policy makers, program planner, and implementers to improve maternal and neonatal outcomes. This figure is in line with findings of studies held in Sudan and Tanzania [41, 42]. But the finding is much higher than systematic review done in Iran and CDC estimation and studies conducted in Bangladesh, South Africa, Cameroon, and Saudi Arabia [3, 43–47]. However, the figure of this review is much lower than result of studies conducted in Egypt, Pakistan, and Libya which was 32%, 23.9%, and 30%, respectively [48–50].

In addition to estimating the pooled burden of UTI, this meta-analysis also identified factors to be associated with the pooled prevalence of UTI among pregnant women in Ethiopia. Among factors evaluated, only family monthly income, parity, history of catheterization, and history of UTI were significantly associated factors with the overall pooled prevalence of UTI among pregnant women in Ethiopia.

The odds of UTI among pregnant women whose family income was less than 1000ETB were higher than their counterparts. This figure is in line with studies conducted in Egypt and Pakistan [2, 49]. This could be evidenced that pregnant women with low economic status were majorly exposed to malnutrition in turn had impact on immunity status. Parity was also another factor significantly that increased the odds of UTI during pregnancy. The likelihood of UTI was higher among multipara pregnant women than primipara and nulliparous pregnant women. This finding is line with result of studies conducted in Nigeria, Iran, and Pakistan [2, 51, 52].

The association between multiparity and UTI is due to profound physiologic changes affecting the entire urinary tract during pregnancy has a significant impact on the natural history of UTI during gestation [53]. These changes vary from patient to patient and are more likely to occur in women who have pregnancies in rapid succession. Furthermore, the anatomical relationship of the female urethra to the vagina makes it liable to trauma during childbirth [54].

In addition, previous history of UTI was a significant factor associated with UTI among pregnant women. The odds of UTI among pregnant women who had history of UTI were higher than their counterparts. This result was in agreement with studies conducted in Pakistan, Qatar, Philippines [2, 53, 55], and Saudi Arabia [44]. This may be evidenced by the risk of developing resistance strains increased among pregnant women who had previous history of UTI.

Once more, this review revealed that the odds of UTI among pregnant women who had previous history of catheterization were higher than their counterparts. This finding is supported with studies conducted in Korea, Israel, and Nigeria [56–58]. This might be due to catheterization is an invasive procedure and could induce urethral mucosa injury. It can also lead to the introduction of bacterial organism to the bladder which induces haematogenous bacterial spread due to failure in infection prevention or poor aseptic technique which can be responsible for recurrent UTI [4, 59]. Generally, this concrete evidences will have positive influential impact to improve maternal and neonatal health in terms of alleviating this high burden of UTI. In addition, this evidence will be used as baseline for healthy policy makers, planners, and implementers.

### 4.1. Study Limitation

All included studies were cross-sectional study design in which the result might potentially be affected by confounding variables and difficult to establish temporal relationship between the outcome and exposure variables. In addition, the meta-analysis did not include all regions and administrative city which only include four regions and two administrative city of the country. Therefore, further country-based studies to assess other confounding factors related to health service-related factors in terms of quality, health policy factors, and health caregiver-related factors are recommended.

## 5. Conclusion

The overall pooled estimate of UTI among pregnant women in Ethiopia was higher than Communicable Disease Control (CDC) estimation which was 8%. Both sociodemographic, medical, and obstetric related factors which can be prevented affect the pooled prevalence of UTI among pregnant women. Family monthly income < 1000ETB, multipara, previous history of catheterization, and history of UTI were factors increased burden of UTI during pregnancy. These findings indicated the need for interventions. So, strategies targeting in economic reforms and universal access of family planning were needed. In addition, standardized prenatal care service as recommended to identify those risk factors early should be addressed by the Ministry of Health and its stakeholders to alleviate this high prevalence of UTI during pregnancy and its complications.

## Figures and Tables

**Figure 1:** PRISMA flow diagram of included studies to estimate the pooled *prevalence* of UTI and its associated factors among pregnant women in Ethiopia from 2007 to 2018.

**Figure 2:** Forest plot of the pooled prevalence of UTI and its associated factors among pregnant women in Ethiopia from 2007 to 2018.

**Figure 3:** Meta funnel presentation of the pooled prevalence of UTI and its associated factors among pregnant women in Ethiopia from 2007 to 2018.

**Figure 4:** Forest plots which describe association between maternal age, marital status, education and income, and UTI among pregnant women in Ethiopia from 2007 to 2018.

**Figure 5:** Forest plots which describe association of history of UTI, anemia, HIV status, occupation, and residence with UTI among pregnant women in Ethiopia from 2007 to 2018.

**Figure 6:** Forest plots which describe association of history of catheterization, parity, and gestational age with UTI among pregnant women in Ethiopia from 2007 to 2018.

**Table 1:** Descriptive summary of 14 studies included in the meta-analysis of pooled *prevalence* of UTI and its associated factors among pregnant women in Ethiopia from 2007 to 2018.

Author	Publication year	Region	E. coli	GNB	GPB	Sampling technique	Mean age	RR (%)	Sample size	Prevalence (%)	JBI score
Derese et al.	2016	Dire Dawa	34.6	73	27	Consecutive	-	100%	186	14	5
Derbie et al.	2018	Amhara	11.1	25.9	74.1	Consecutive	26.8	100%	234	11.5	5
Ali et al.	2018	Amhara	31	36.2	63.8	Consecutive	26.5	100%	358	15.6	6
Alemu et al.	2012	Amhara	47.5	67.5	32.5	SyRS	26	100%	385	10.4	8
Ferede et al.	2012	Amhara	41.5	58.3	41.7	Consecutive	28	95%	200	12	6
Tsegay et al.	Unpub	Tigray	30	60	40	Consecutive	25	100%	168	11.9	5
Taye et al.	2018	SNNP	27.3	-	-	SyRS	-	100%	169	26	8
Tadesse et al.	2018	Tigray	34.6	64.1	35.9	Consecutive	26	100%	259	21.2	7
Tadesse E et al.	2014	SNNP	26.1	49	51	Consecutive	26.13	100%	244	18.8	6
Tadesse A et al.	2007	Amhara	47	-	-	Consecutive	26	96%	173	9.8	5
Nisha et al.	2015	Oromo	37.3	-	-	Consecutive	25.7	100%	367	26.6	7
Zebene et al.	Unpub	AA	44.4	-	-	Consecutive	27	100%	424	14.9	5
Asefa et al.	2008	AA	44	60	40	Consecutive	-	100%	414	11.6	5
Emiru et al.	2013	Amhara	-	-	-	Consecutive	-	100%	367	-	7

**Table 2:** Criteria used for scoring of risk bias assessment tool of included articles for the estimation of pooled prevalence of UTI and its associated factors among pregnant women in Ethiopia from 2007 to 2018.

Criteria	Bias score		
	Low risk	Medium risk	High risk
Representation	12 studies	-	2 studies
Sampling	2 studies	-	12 studies
Random selection	4 studies	-	10 studies
Nonresponse bias	14 studies	-	-
Data collection	14 studies	-	-
Case definition	14 studies	-	-
Reliability and validity of study tool	10 studies	-	4 studies
Method of data collection	10 studies	-	4 studies
Prevalence period	14 studies	-	-
Numerator and denominator	14 studies	-	-
Summary assessment	10 studies	-	4 studies

**Table 3:** Subgroup analysis which describes pooled burden of UTI and its associated factors among pregnant women in Ethiopia from 2007 to 2018.

Subgroup		No. of studies	Prevalence (95% CI)	Heterogeneity statistics	*I* ^2^	*p* value
Region	Amhara	5	11.61 (9, 13)	3.03	0.0	0.553
	Tigray	2	16.37 (7, 25)	5.59	82.1	0.018
	SNNPR	2	22.26 (15, 29)	2.70	62.9	0.101
	AA	2	13.09 (9, 16)	0.82	0.0	0.366
	Others	2	20.14 (7, 32)	8.95	88.1	0.003

Publication year	Before 2015	5	12.19 (9, 15)	6.79	41.1	0.143
	2015 & above	6	18.88 (13, 23)	24.13	79.3	<0.001
	Unpublished	2	13.27 (9, 16)	0.67	0.0	0.412

Sampling technique	Consecutive	11	14.92 (12, 17)	30.01	66.7	0.001
	Systematic random	2	18.03 (2, 33)	15.12	92.1	<0.001

Sample size	<250	7	14.51 (10, 18)	22.00	72.1	0.001
	>250	6	16.4 (11, 21)	22.25	77.5	<0.001

**Table 4:** Metaregression for the included studies to identify source of heterogeneity for the pooled prevalence of UTI and its associated factors among pregnant women in Ethiopia from 2007 to 2018.

Variables	Coefficients	*p* value
Study year	-0.126	0.078
Sample size	-0.019	0.602
Mean age	0.91	0.532
Region		
Amhara	-8.60	0.056
SNNPR	1.53	0.758
Tigray	-3.94	0.424
AA	-7.25	0.144

## Data Availability

Data will be available from the corresponding author upon reasonable request.

## Abbreviations

AA: Addis Ababa
CDC: Communicable Disease Control
SNNP: South Nation and Nationality peoples
UTI: Urinary tract infection
WHO: World Health Organization.

## References

[1] Hill J. B., Sheffield J. S., McIntire D. D., Wendel G. D. (2005). Acute pyelonephritis in pregnancy. *Obstetrics & Gynecology*.

[2] Haider G., Zehra N., Munir A. A., Haider A. (2010). Risk factors of urinary tract infection in pregnancy. *JPMA The Journal of the Pakistan Medical Association*.

[3] Delzell J. E., LeFevre M. (2000). Urinary tract infections during pregnancy. *American Family Physician*.

[4] Storme O., Tiran Saucedo J., Garcia-Mora A., Dehesa-Dávila M., Naber K. G. (2019). Risk factors and predisposing conditions for urinary tract infection. *Therapeutic Advances in Urology*.

[5] Kalinderi K., Delkos D., Kalinderis M., Athanasiadis A., Kalogiannidis I. (2018). Urinary tract infection during pregnancy: current concepts on a common multifaceted problem. *Journal of Obstetrics and Gynaecology*.

[6] Hooton T. M. (2012). Uncomplicated urinary tract infection. *New England Journal of Medicine*.

[7] Glaser A. P., Schaeffer A. J. (2015). Urinary tract infection and bacteriuria in pregnancy. *Urologic Clinics*.

[8] Dimetry S. R., El-Tokhy H. M., Abdo N. M., Ebrahim M. A., Eissa M. (2007). Urinary tract infection and adverse outcome of pregnancy. *The Journal of the Egyptian Public Health Association*.

[9] Yan L., Jin Y., Hang H., Yan B. (2018). The association between urinary tract infection during pregnancy and preeclampsia: a meta-analysis. *Medicine*.

[10] Valkenburg-van den Berg A. W., Sprij A. J., Dekker F. W., Dörr P. J., Kanhai H. H. (2009). Association between colonization with group BStreptococcusand preterm delivery: a systematic review. *Acta Gynecologica Scandinavica*.

[11] Gilbert N. M., O’brien V. P., Hultgren S., Macones G., Lewis W. G., Lewis A. L. (2013). Urinary tract infection as a preventable cause of pregnancy complications: opportunities, challenges, and a global call to action. *Global advances in health and medicine*.

[12] Kazemier B. M., Koningstein F. N., Schneeberger C. (2015). Maternal and neonatal consequences of treated and untreated asymptomatic bacteriuria in pregnancy: a prospective cohort study with an embedded randomised controlled trial. *The Lancet Infectious Diseases*.

[13] Mazor-Dray E., Levy A., Schlaeffer F., Sheiner E. (2009). Maternal urinary tract infection: is it independently associated with adverse pregnancy outcome?. *The Journal of Maternal-Fetal & Neonatal Medicine*.

[14] Schieve L. A., Handler A., Hershow R., Persky V., Davis F. (1994). Urinary tract infection during pregnancy: its association with maternal morbidity and perinatal outcome. *American Journal of Public Health*.

[15] ACOG (2012). *Guidelines for Perinatal Care*.

[16] Whitehead N. S., Callaghan W., Johnson C., Williams L. (2009). Racial, ethnic, and economic disparities in the prevalence of pregnancy complications. *Maternal and Child Health Journal*.

[17] Alvarez J. R., Fechner A. J., Williams S. F., Ganesh V. L., Apuzzio J. J. (2010). Asymptomatic bacteriuria in pregestational diabetic pregnancies and the role of group B Streptococcus. *American Journal of Perinatology*.

[18] Wing D. A., Fassett M. J., Getahun D. (2014). Acute pyelonephritis in pregnancy: an 18-year retrospective analysis. *American Journal of Obstetrics and Gynecology*.

[19] Tadesse A., Negash M., Ketema L. (2007). Asymtomatic bacteriuria in pregnancy: assesment of prevlence, microbial agents and ther antimicrobial sensitivty pattern in Gondar Teaching Hospital, north west Ethiopia. *Ethiopian Medical Journal*.

[20] Nisha A. K., Etana A. E., Tesso H. (2015). Prevalence of asymptomatic bacteriuria during pregnancy in Adama city, Ethiopia. *Int J Microbiol Immunol Res*.

[21] Alemu A., Moges F., Shiferaw Y. (2012). Bacterial profile and drug susceptibility pattern of urinary tract infection in pregnant women at University of Gondar Teaching Hospital, Northwest Ethiopia. *BMC Research Notes*.

[22] Ali I. E., Gebrecherkos T., Gizachew M., Menberu M. A. (2018). Asymptomatic bacteriuria and antimicrobial susceptibility pattern of the isolates among pregnant women attending Dessie referral hospital, Northeast Ethiopia: a hospital-based cross-sectional study. *Turkish Journal of Urology*.

[23] Assefa A., Asrat D., Woldeamanuel Y., Abdella A., Melesse T. (2008). Bacterial profile and drug susceptibility pattern of urinary tract infection in pregnant women at Tikur Anbessa Specialized Hospital Addis Ababa, Ethiopia. *Ethiopian Medical Journal*.

[24] Demilie T., Beyene G., Melaku S., Tsegaye W. (2014). Diagnostic accuracy of rapid urine dipstick test to predict urinary tract infection among pregnant women in Felege Hiwot Referral Hospital, Bahir Dar, North West Ethiopia. *BMC Research Notes*.

[25] Derese B., Kedir H., Teklemariam Z., Weldegebreal F., Balakrishnan S. (2016). Bacterial profile of urinary tract infection and antimicrobial susceptibility pattern among pregnant women attending at Antenatal Clinic in Dil Chora Referral Hospital, Dire Dawa, Eastern Ethiopia. *Therapeutics and Clinical Risk Management*.

[26] Emiru T., Beyene G., Tsegaye W., Melaku S. (2013). Associated risk factors of urinary tract infection among pregnant women at Felege Hiwot Referral Hospital, Bahir Dar, North West Ethiopia. *BMC Research Notes*.

[27] Ephrem T. (2014). *Bacterial profile and drug susceptibility pattern of urinary tract infection in pregnant women attending antenatal care at Mekelle Hospital, Mekelle, Northern Ethiopia. Un-publish*.

[28] Ferede G., Yismaw G., Wondimeneh Y., Sisay Z. (2012). The prevalence and antimicrobial susceptibility pattern of bacterial uropathogens isolated from pregnant women. *Eur J Exp Biol*.

[29] Habteyohannes A. D., Mekonnen D., Abate E., Tadesse S., Birku T., Biadglegne F. (2018). Bacterial isolates and their current drug susceptibility profile from urine among asymptomatic pregnant women attending at a Referral Hospital, Northwest Ethiopia; cross-sectional study. *Ethiopian Journal of Reproductive Health*.

[30] Tadesse E., Teshome M., Merid Y., Kibret B., Shimelis T. (2014). Asymptomatic urinary tract infection among pregnant women attending the antenatal clinic of Hawassa Referral Hospital, Southern Ethiopia. *BMC Research Notes*.

[31] Tadesse S., Kahsay T., Adhanom G., Kahsu G., Legese H., Derbie A. (2018). Prevalence, antimicrobial susceptibility profile and predictors of asymptomatic bacteriuria among pregnant women in Adigrat General Hospital, Northern Ethiopia. *BMC Research Notes*.

[32] Taye S., Getachew M., Desalegn Z., Biratu A., Mubashir K. (2018). Bacterial profile, antibiotic susceptibility pattern and associated factors among pregnant women with Urinary Tract Infection in Goba and Sinana Woredas, Bale Zone, Southeast Ethiopia. *BMC Research Notes*.

[33] Zebene W. (2019). *Urinary Tract Infection, Drug Resistance Profile and Fetal Outcomes among Pregnant Women in Two Health Centers and Tikur Anbessa Specialized Hospital, Addis Ababa*.

[34] Liberati A., Altman D. G., Tetzlaff J. (2009). The PRISMA statement for reporting systematic reviews and meta-analyses of studies that evaluate health care interventions: explanation and elaboration. *Journal of Clinical Epidemiology*.

[35] Munn Z., Moola S., Lisy K., Riitano D. (2014). *The Joanna Briggs institute reviewers’ manual. The systematic review of prevalence and incidence data*.

[36] Hoy D., Brooks P., Woolf A. (2012). Assessing risk of bias in prevalence studies: modification of an existing tool and evidence of interrater agreement. *Journal of Clinical Epidemiology*.

[37] Huedo-Medina T. B., Sánchez-Meca J., Marín-Martínez F., Botella J. (2006). Assessing heterogeneity in meta-analysis: Q statistic or ^I²^ index?. *Psychological Methods*.

[38] Rendina-Gobioff G. (2006). *Detecting publication bias in random effects meta-analysis*.

[39] Getaneh T., Negesse A., Chane J. (2019). *Premarital sexual practice and its associated factors in Ethiopia*.

[40] Gebre-Selassie S. (1998). Asymptomatic bacteriuria in pregnancy: epidemiological, clinical and microbiological approach. *Ethiopian Medical Journal*.

[41] Masinde A., Gumodoka B., Kilonzo A., Mshana S. (2009). Prevalence of urinary tract infection among pregnant women at Bugando Medical Centre, Mwanza, Tanzania. *Tanzania Journal of Health Research*.

[42] Hamdan H. Z., Ziad A. H. M., Ali S. K., Adam I. (2011). Epidemiology of urinary tract infections and antibiotics sensitivity among pregnant women at Khartoum North Hospital. *Annals of Clinical Microbiology and Antimicrobials*.

[43] Azami M., Jaafari Z., Masoumi M. (2019). The etiology and prevalence of urinary tract infection and asymptomatic bacteriuria in pregnant women in Iran: a systematic review and meta-analysis. *BMC Urology*.

[44] Faidah H. S., Ashshi A. M., Abou El-Ella G. A., Al-Ghamdi A. K., Mohamed A. M. (2013). Urinary tract infections among pregnant women in Makkah, Saudi Arabia. *Biomedical And Pharmacology Journal*.

[45] Uddin M. N., Khan T. (2016). Prevalence of urinary tract infection among pregnant women at Ibrahim Iqbal Memorial Hospital, Chandanaish, Bangladesh. *Am J Clin Med Res*.

[46] Siemefo Kamgang F. D. P., Maise H. C., Moodley J. (2016). Pregnant women admitted with urinary tract infections to a public sector hospital in South Africa: are there lessons to learn?. *Southern African Journal of Infectious Diseases*.

[47] Nguefack C. T., Ebongue C. O., Chokotheu C. N., Ewougo C. E., Njamen T. N., Mboudou E. (2019). Clinical presentation, risk factors and pathogens involved in bacteriuria of pregnant women attending antenatal clinic of 3 hospitals in a developing country: a cross sectional analytic study. *BMC Pregnancy and Childbirth*.

[48] Sheikh M. (2000). *Incidence of Urinary Tract Infection during Pregnancy*.

[49] Shaheen H. M., Farahat T. M., NAE-H H. (2016). Prevalence of urinary tract infection among pregnant women and possible risk factors. *Menoufia Medical Journal*.

[50] Tamalli M., Bioprabhu S., Alghazal M. (2013). Urinary tract infection during pregnancy at Al-khoms, Libya. *Int J Med Med Sci*.

[51] Okonko I., Ijandipe L., Ilusanya O. (2009). Incidence of urinary tract infection (UTI) among pregnant women in Ibadan, South-Western Nigeria. *African Journal of Biotechnology*.

[52] Enayat K., Fariba F., Bahram N. (2008). Asymptomatic bacteriuria among pregnant women referred to outpatient clinics in Sanandaj, Iran. *International Braz J Urol*.

[53] Nandy P., Thakur A., Ray C. (2007). Characterization of bacterial strains isolated through microbial profiling of urine samples. *On Line J Biol Sci*.

[54] Kolawole A., Kolawole O., Kandaki-Olukemi Y., Babatunde S., Durowade K., Kolawole C. (2009). Prevalence of urinary tract infections (UTI) among patients attending Dalhatu Araf Specialist Hospital, Lafia, Nasarawa state, Nigeria. *International journal of medicine and medical sciences*.

[55] Aseel M. T., Al-Meer F. M., Al-Kuwari M. G., Ismail M. F. S. (2009). Prevalence and predictors of asymptomatic bacteriuria among pregnant women attending primary health care in Qatar. *WORLD FAMILY MEDICINE*.

[56] Onwuezobe I., Orok F. (2015). Associated risk factors of asymptomatic urinary tract infection among pregnant women attending antenatal care in a secondary health care facility in a south-south Nigerian City. *International Journal of Current Microbiology and Applied Sciences*.

[57] Lee S.-E., Kim K.-T., Park Y.-S., Kim Y.-B. (2010). Association between asymptomatic urinary tract infection and postoperative spine infection in elderly women: a retrospective analysis study. *Journal of Korean Neurosurgical Society*.

[58] Vardi M., Kochavi T., Denekamp Y., Bitterman H. (2012). Risk factors for urinary tract infection caused by Enterobacteriaceae with extended spectrum beta-lactamase resistance in patients admitted to internal medicine departments. *Sat*.

[59] Akerele P., Abhulimen F., Okonofua J. (2001). Prevalence of asymptomatic bacteriuria among pregnant women in Benin City, Nigeria. *Journal of Obstetrics and Gynaecology*.

